# Racial and Ethnic Disparities in Health Outcomes Among Long-Term Survivors of Childhood Cancer: A Scoping Review

**DOI:** 10.3389/fpubh.2021.741334

**Published:** 2021-10-29

**Authors:** Tegan J. Reeves, Taylor J. Mathis, Hailey E. Bauer, Melissa M. Hudson, Leslie L. Robison, Zhaoming Wang, Justin N. Baker, I-Chan Huang

**Affiliations:** ^1^Department of Epidemiology and Cancer Control, St. Jude Children's Research Hospital, Memphis, TN, United States; ^2^Department of Oncology, St. Jude Children's Research Hospital, Memphis, TN, United States; ^3^Department of Computational Biology, St. Jude Children's Research Hospital, Memphis, TN, United States

**Keywords:** childhood cancer survivor, ethnicity, health disparities, health outcomes, race

## Abstract

The five-year survival rate of childhood cancer has increased substantially over the past 50 yr; however, racial/ethnic disparities in health outcomes of survival have not been systematically reviewed. This scoping review summarized health disparities between racial/ethnic minorities (specifically non-Hispanic Black and Hispanic) and non-Hispanic White childhood cancer survivors, and elucidated factors that may explain disparities in health outcomes. We used the terms “race”, “ethnicity”, “childhood cancer”, “pediatric cancer”, and “survivor” to search the title and abstract for the articles published in PubMed and Scopus from inception to February 2021. After removing duplicates, 189 articles were screened, and 23 empirical articles were included in this review study. All study populations were from North America, and the mean distribution of race/ethnicity was 6.9% for non-Hispanic Black and 4.5% for Hispanic. Health outcomes were categorized as healthcare utilization, patient-reported outcomes, chronic health conditions, and survival status. We found robust evidence of racial/ethnic disparities over four domains of health outcomes. However, health disparities were explained by clinical factors (e.g., diagnosis, treatment), demographic (e.g., age, sex), individual-level socioeconomic status (SES; e.g., educational attainment, personal income, health insurance coverage), family-level SES (e.g., family income, parent educational attainment), neighborhood-level SES (e.g., geographic location), and lifestyle health risk (e.g., cardiovascular risk) in some but not all articles. We discuss the importance of collecting comprehensive social determinants of racial/ethnic disparities inclusive of individual-level, family-level, and neighborhood-level SES. We suggest integrating these variables into healthcare systems (e.g., electronic health records), and utilizing information technology and analytics to better understand the disparity gap for racial/ethnic minorities of childhood cancer survivors. Furthermore, we suggest national and local efforts to close the gap through improving health insurance access, education and transportation aid, racial-culture-specific social learning interventions, and diversity informed training.

## Introduction

The shifting racial/ethnic makeup of the population indicates that in as early as 2045 the United States (US) will become a “minority majority population” country (1). By 2060, non-White individuals will make up more than 60% of the population (2). Racial/ethnic disparities in health are the race- and ethnicity-specific illnesses, injuries, or mortality (3) that disproportionately impact the marginalized groups. The growing diversity of the US population will be accompanied by growing health disparities.

Health equity is considered one of the four basic human rights (3), yet determinants of the inequity and effective implementation strategies to improve racial/ethnic disparity in health outcomes are still limited. Although life expectancy of the US general population has steadily increased since the 1950s in the US, non-Hispanic Black individuals have a 40% higher overall mortality rates (4) and non-Hispanic Black and Hispanic populations have a higher burden of chronic health conditions (e.g., cancer, heart disease, diabetes) (5) compared to non-Hispanic White individuals. In addition, minority populations often have lower healthcare utilization and access to quality care (6). In the context of oncology, health disparities in the US are significantly different in the rates of cancer screening, incidence, survival, treatment-related complications, and quality-of-life (7). Although the 5-yr relative cancer survival rates of childhood cancer have reached 94% among the child and 85% among adolescent survivors (8), there is evidence of lower patient-reported outcomes and survival rates (9–11) in minority vs. non-Hispanic White survivors. Furthermore, the mechanisms behind these disparities are understudied.

While scholars have yet to agree on specifics, it is clear that health disparities are influenced by multiple factors. Some argue that socioeconomic status (SES) is a stronger determinant of health outcomes than race *per se* (12). Others suggest that cultural (13) or population-level factors (14) contribute to health disparities in childhood cancer survivors. Neighborhoods with a higher proportion of Black or Hispanic residents are associated with higher poverty due to a lack in community investment and built environments (i.e., fast food restaurants, liquor stores, lack of green space) which decrease the opportunities for healthy eating and exercises (15). Disadvantaged neighborhood conditions (e.g., high crime rate, poor community support, collective efficacy or social capital) have shown elevated mortality through the mechanisms of practicing health behaviors (16).

The main objective of this study was to summarize the evidence of racial/ethnic disparities in health outcomes for survivors of childhood cancer based on a scoping review of previously published literature. We focused on race/ethnicity as the primary variable determining disparities in health outcomes, and viewed SES factors as confounding or mediating variables that explain the associations between race/ethnicity and health outcomes. This is because the vast majority of the studies selected are based on the cross-sectional design, and the true effect of SES factors on health outcomes cannot be determined (e.g., survivors having lower incomes may develop worse chronic health conditions, and worse health conditions may further lower survivors' incomes). Specifically, we aimed to elucidate the role that personal/family/community-level SES factors alongside other demographic and clinical factors might play to explain the associations between race/ethnicity and health outcomes. Based on these findings, we made recommendations toward improving health disparities for minority childhood cancer survivors, especially by identifying modifiable social determinants of health using information technology, integrating social determinant information into healthcare systems, and suggesting potential interventions for health outcomes improvement.

## Methods

In line with our aims, a scoping review was performed to aggregate evidence from empirical studies. Scoping reviews are particularly useful for complex/diverse issues (17) such as race/ethnicity, and generally precede systematic and meta-analyses (18).

### Article Selection and Screening Process

We performed a literature search process according to the Preferred Reporting Items for Systematic Reviews and Meta-Analyses Extension for Scoping Reviews (PRISMA-ScR) (19). Two independent investigators researched the title and abstract for articles published between inception and February 2021 in the PubMed and Scopus using the terms “race”, “ethnicity”, “childhood cancer”, “pediatric cancer”, and “survivor”. In addition, the search was limited to articles published in the English language and available in full-text. The initial search yielded 26 articles from PubMed and 173 articles from Scopus. After removing duplicates, a combined total of 189 articles were prepared for screening.

Two independent investigators screened the articles for inclusion if these articles included the following criteria: health disparity (i.e. difference in outcome based on race/ethnicity), health outcomes/late effects, and any age range of the survivorship stage. We excluded articles if they met the following criteria: not reporting health outcomes/late effects (90 articles), race/ethnicity listed but only in descriptive statistics (64 articles), no full-text available (4 articles), and absence of IRB approval or otherwise proof of rigor (e.g., qualitative, opinion, review, briefs, and meta-analysis; 6 articles). In addition, two Swiss articles were removed from subsequent review because they did not include non-Hispanic Black or Hispanic survivors. We included two articles that use the term “non-White” (i.e., a combined concept for non-Hispanic Black and Hispanic) into our review.

### Data Charting

We extracted data from each article according to the study design, race/ethnicity, health outcomes, and risk modulators of racial/ethnic disparity in health outcomes. We focused on marginalized/minoritized (20). US categories of non-Hispanic Black and Hispanic, and reported its association with health disparity.

We classified health outcomes of childhood cancer survivors by four distinct categories: (1) healthcare utilization, (2) patient-reported outcomes, (3) chronic health conditions, and (4) survival rates. For counting health outcomes of interest, if studies reported outcomes in more than one category, these studies were listed in different, separate outcome categories. Healthcare utilization outcomes included the concept of healthcare self-efficacy, initial and follow-up care visits, contact with general or cancer-specific healthcare providers, and use of hospital services. Patient-reported outcomes included the concept of health-related quality of life, symptom presence or severity, adaptive functioning, and post-traumatic stress. Chronic health conditions represented individual health conditions (e.g., diabetes) or organ system-based condition groups (e.g., endocrine). Survival outcomes were categorized as all-cause or condition-specific survival rates. In addition, we reported the factors used to explain racial/ethnic disparities in health outcomes per the rationale of the articles or statistical modeling process (e.g., the mediating effects from the path analysis and covariate-adjustment or interaction effects from the standard regression models).

## Results

### Characteristics of the Selected Articles

Figure 1 presents the PRISMA flow diagram for the process of article selection. Of 185 full-text articles initially identified, 23 articles which met the inclusion/exclusion criteria were selected into full review and data extraction. Table 1 summarizes the characteristics of the 23 selected articles, published between 2002 and 2020. All study populations included in the 23 articles were from North America. A majority (52%) of the selected articles were based on the US National Cancer Institute-funded Childhood Cancer Survivorship Study or the US Surveillance, Epidemiology, and End Results program (SEER). The size of the samples ranged from under 100 (5 articles) to over 10,000 (6 articles). The age range of survivors included in the 23 articles varied from adolescents (7 articles) and young adults (5 articles) to adults (5 articles) or all ages (6 articles). The distribution of race/ethnicity was calculated and presented as percentage with non-Hispanic White as the reference group (see Table 1). The average percentages were 6.9% for non-Hispanic Black and 4.5% for Hispanic, which were smaller compared to 13.4% for non-Hispanic Black and 18.5% for Hispanic in the general US population (45). Data abstracted from the selected studies were all cross-sectional in nature. A variety of statistical techniques were used to test the statistical difference and suggest the influential factors. The most used methods included multivariate modeling (13 articles) and ratio-based models [e.g., odds ratio (3 articles), proportional hazards (2 articles), or standardized ration (3 articles)]; other methods included analysis of covariance and flexible parameters model.

**Figure 1:** PRISMA diagram of study selection. Adapted from (21).

**Table 1:** Characteristics of studies included in the scoping review.

**References**	**Sample size**	**Age (years)**	**Population**	**Race/Ethnicity (%)**	**Health outcome category**	**Specific health outcomes**
Armstrong et al. (22)	*N =* 26443	0–18	SEER	NHB (8.8); H (14.4)	Survival rates	All-cause mortality; non-recurrence/non-external mortality
Arpawong et al. (23)	*N =* 94	11–21	Treatment Center	Hispanic (English 27.6; ESL, 19.1)	Patient-reported outcomes	Post-traumatic growth, post-traumatic stress
Barrera et al. (24)	*N =* 74	8–16^*^	Canadian Children's	Black (5.4)	Patient-reported outcomes	Quality of life and emotional quality of life
Berkman et al. (25)	*N =* 164316	0–34^*^	SEER	Black (10.7)	Chronic health conditions and survival rates	Cardiovascular conditions, overall mortality
Castellino et al. (26)	*N =* 8767	≥18	CCSS	Hispanic (15.6)	Healthcare utilization, patient-reported outcomes	Screening, mental health
Choudhary et al. (27)	*N =* 484	2–36^**^	Sloan Kettering	Black (12.1); Hispanic (15.6)	Chronic health conditions	Vitamin-D deficiency i.e. chemiluminescent assay
Daly et al. (28)	*N =* 866	>6	CHOA	48.5% Non-White	Healthcare utilization	Initial visit
Gance-Cleveland et al. (29)	*N =* 321	6–21^*^	Survivor Clinic	Black (2.4); Hispanic (29.9)	Chronic health conditions	Obesity
Kehm et al. (30)	*N =* 31866	0–19^*^	SEER	NHB (11.8); Hispanic (31.5)	Survival rates	Overall survival
Liu et al. (31)	*N =* 13841	8–58	CCSS	NHB (5); Hispanic (5.4)	Survival rates and chronic health conditions	Cardiovascular condition, overall mortality
Lu et al. (32)	*N =* 10362	18–38	CCSS	NHB (4.3); Hispanic (1.9)	Patient-reported outcomes	Pain
Meeske et al. (33)	*N =* 86	8–18^*^	CHLA	Hispanic (48%)	Patient-reported outcomes	Total and psychosocial function
Meeske et al. (34)	*N =* 139	14–25^**^^+^	CSP	Hispanic (US, 12.9; foreign born 43.8)	Patient-reported outcomes	Parent post-traumatic stress, depression
Milam et al. (35)	*N =* 193	14–25^**^	LA SEER	Hispanic (54.4)	Healthcare utilization	Follow-up care
Miller et al. (36)	*N =* 193	≥15	LA SEER	Hispanic (54.4)	Healthcare utilization	Healthcare self-efficacy
Miller et al. (37)	*N =* 193	≥15^*^	LA SEER	Hispanic (54.4)	Healthcare utilization	Information seeking
Oikonomou et al. (38)	*N =* 88,418	0–19^*^	SEER	Black (10.7); Other (8.1)	Chronic health conditions	Cardiovascular condition
Raghubar et al. (39)	*N =* 114	5–21^*^^+^	CHLA	Hispanic (29.8); Other (19.2)	Patient-reported outcomes	Adaptive functioning
Samaan et al. (40)	*N =* 5956	0–19^**^	SEER	Non-White (17.8)	Survival rates	Mortality to incidence ratio and relative survival trend
Santacroce et al. (41)	*N =* 15	37.9 ^+^^#^	Clinic	Black (33.3)	Patient-reported outcomes	Uncertainty, anxiety, stress
Tobin et al. (42)	*N =* 235	14–25	CSP	Hispanic (56.2)	Patient-Reported outcome	Post-traumatic growth
Wasilewski-Masker et al. (43)	*N =* 519	12.1^#^	CHOA	Black (14)	Chronic health condition	Severity of symptoms (CTCEA)
Zebrack et al. (44)	*N =* 6425	≥18	CCSS	Non-White (6.4)	Patient-reported outcomes	Positive impact

* *Less than 5 years since last treatment;*

** *No information on years since last treatment;*

+ *Parent responses;*

# *Mean age reported in years at survey/assessment; Reference Group: Non-Hispanic White*.

*CCSS, Childhood Cancer Survivor Study; CHLA, Children's Hospital of Los Angeles; CHOA, Childhood Healthcare of Atlanta; CHOC, Children's Hospital of Orange County; CSP, Los Angeles Cancer Surveillance Program; SEER, Surveillance Epidemiology and End Results Program*.

### Disparities in Healthcare Utilization

Five articles reported racial/ethnic disparities in healthcare utilization (Table 2). The type of healthcare utilization disparities reported for non-Hispanic Black survivors included general medical contact (26) and an initial survivorship visit (28). The type of healthcare utilization disparities reported for Hispanic survivors included general medical contact (26), a cancer center visit (26), the use of follow-up care (35), health-care self-efficacy, defined as perceived control and confidence in managing healthcare (36), and seeking information from a hospital (37) or from family members (37). Across the articles, risk modulators included in analytic models for healthcare utilization disparities included clinical factors (diagnosis, treatment), individual characteristics (age, sex, depressive symptoms, post-traumatic growth, self-efficacy), individual-/family-level SES (educational attainment, household income, health insurance coverage), and social/contextual factors (support, family influence).

**Table 2:** Factors influencing disparities in healthcare utilization for childhood cancer survivors by race/ethnicity.

**Source**	**Risk modulators**	**Results of unadjusted models**	**Results of adjusted models**	**Interpretation of findings**
**NON-HISPANIC BLACK**				
(26)	SES (insurance, education, household income), age, diagnosis	**OR = 0.6; 95% CI: 0.5–0.9**	OR = 0.7; 95% CI: 0.5–1.0 (males)	Lower general medical contact attenuated by risk modulators.
(26)	SES (insurance, education, household income), age, diagnosis		**OR = 0.5; 95% CI: 0.3–0.7 (females)**	Lower general medical contact accounting for risk modulators.
(28)	Gender, age, treatment factors (year and age of diagnosis, diagnosis, therapy subsequent event), and logistic factors (insurance, distance from clinic)	**HR = 0.77, 95% CI: 0.64–0.94**	**HR= 0.64, 95% CI: 0.52–0.79**	Less likely to have initial survivorship visit.
**HISPANIC**				
(26)	SES (insurance, education, household income), age, diagnosis		**OR = O.6; 95% CI: 0.4–0.8**	Lower general medical contact accounting for risk modulators.
(26)	SES (insurance, education, household income), age, diagnosis		OR = 1.7, 95% CI: 1.2–2.3 (males) OR = 1.5, 95% CI: 1.1–2.0 (females)	More likely to visit cancer center accounting for risk modulators.
(35)	Age, sex, social support, family influence, post traumatic growth, depressive symptoms, treatment, self-efficacy	OR = 0.55, 95% CI: 0.25–1.21, *p =* 0.17	**OR = 0.33, 95% CI: 0.11−0.96**, ***p =*** **0.03**	Less likely to report previous use of follow-up care after accounting for risk modulators.
(36)	Age, sex, social support, family influence, post traumatic growth, depressive symptoms, treatment, self-efficacy	β = −0.38 (0.19), *p* < 0.1	**β = −0.42 (0.20)**, ***p <*** **0.05**	Lower health-care self-efficacy after accounting for risk modulators.
(37)	Age, sex, health insurance	**OR = 2.1, 95% CI: 1.17–3.79**, ***p <*** **0.05**	**OR = 2.52, 95% CI: 1.19–5.30**, ***p <*** **0.05**	Less likely to get information from hospital.
(37)	Age, sex, health insurance	**OR = 0.48, 95% CI: 0.24–0.98**, ***p <*** **0.05**	OR = 0.50, 95% CI: 0.23–1.09, *p* < 0.1	Less likely to get information from family attenuated by risk modulators.

Bold denotes statistical significance with p < 0.05; Reference group Non-Hispanic White or Caucasian; * Reference group listed as Non-Hispanic. SES, Socioeconomic Status; HR, Hazards Ratio; OR, Odd Ratio.

In two articles, inclusion of individual characteristics and individual-/family-level SES in multivariable modeling attenuated the statistical significance for racial/ethnic disparities in healthcare utilization. Specifically, in an odds-ratio model, inclusion of individual-level and family-level SES and individual characteristics (cancer diagnosis and age at the time of study) removed statistical significance of the disparity in general medical contact among non-Hispanic Black male survivors (26). Similarly, inclusion of age, sex, and individual-level SES (i.e., health insurance) removed the statistical significance for receiving less cancer-related information from family members among Hispanic survivors (37). However, two articles found significant racial/ethnic disparity after adjusting for individual characteristics and social contextual factors in the multivariable analyses. Specifically, inclusion of cancer treatment, age, sex, social support, family influence, post-traumatic growth, depressive symptoms, and self-efficacy factors revealed significantly fewer previous receipt of follow-up care among Hispanic survivors compared to non-Hispanic White survivors (35). In addition, inclusion of cancer treatment, age, sex, social support, family influence, post-traumatic growth, and depressive symptoms factors revealed significantly lower healthcare self-efficacy for Hispanic survivors compared to non-Hispanic White survivors (36).

### Disparities in Patient-Reported Outcomes

Nine articles have reported racial/ethnic disparities in patient-reported outcomes (Table 3). The types of patient-reported outcomes assessed for non-Hispanic Black survivors included quality-of-life (24), adverse mental health (26), functional impairment (26), pain or abnormal sensations (32), migraines (32), frequent headaches (32) and parental uncertainty about the child's health (41). The types of patient-reported outcomes assessed for Hispanic survivors included post-traumatic growth (23, 42), psychosocial health (33), quality-of-life (33), school functioning (33), emotional functioning (33), parental post-traumatic stress (34), depression (34), and conceptual, social and practical adaptive functioning (39), pain or abnormal sensations (32), and frequent headaches (32). In addition, the types of patient-report outcomes assessed for non-White survivors included psychosocial functioning (33), quality-of-life (33), school functioning (33), and positive impact of cancer (44). Across the articles, risk modulators included in multivariable modeling comprised clinical factors (diagnosis, treatment), individual characteristics (age, sex, depressive symptoms, post-traumatic stress, optimism, fatigue), individual-/family-level SES (educational attainment, health insurance, household income, parent educational attainment), and social/contextual factors (birthplace, language spoken at home).

**Table 3:** Factors influencing disparities in patient-reported outcomes for childhood cancer survivors by race/ethnicity.

**Source**	**Risk modulators**	**Results of unadjusted models**	**Results of adjusted models**	**Interpretation of findings**
**NON-HISPANIC BLACK**				
(26)	SES (insurance, education, household income), age, diagnosis	OR = 0.8; 95% CI: 0.5–1.2	**OR = 0.6; 95% CI: 0.5–1.0 (females)**	Less adverse mental health after accounting for risk modulators.
(26)	SES (insurance, education, household income), age, diagnosis	**OR =1.7; 95% CI: 1.2–2.5**	OR = 1.2; 95% CI: 0.8–1.8 (females)	Higher functional impairment attenuated by risk modulators.
(32)	None	**HR = 1.91, 95% CI: 1.58–2.30**, ***p <*** **0.001**		Higher reports of pain or abnormal sensation without accounting for risk modulators.
(32)	None	**HR =1.85, 95% CI: 1.54–2.22**, ***p <*** **0.001**		Higher reports of migraines without accounting for risk modulators.
(32)	None	**HR = 1.68, 95% CI: 1.40–2.02**, ***p <*** **0.001**		Higher reports of other frequent headaches without accounting for risk modulators.
(41)		***p <*** **0.001**		Higher parental uncertainty without accounting for risk modulators.
**HISPANIC**				
(32)	None	**HR =1.74, 95% CI: 1.27–2.39**, ***p =*** **0.001**		Higher reports of pain or abnormal sensations without accounting for risk modulators.
(32)	None	**HR = 1.44, 95% CI: 1.06–1.96**, ***p =*** **0.02**		Higher reports of other frequent headaches without accounting for risk modulators.
(23)	Demographics, disease/treatment factors, depressive symptoms, PTSS, optimism, QOL, SES	*p =* 0.52	***p <*** **0.05 (English primary language)**	Lower Post-traumatic Growth (PTG) accounting for risk modulators.
(33)	Diagnosis and fatigue	***p =*** **0.02**	***p <*** **0.01**	Lower psychosocial health after accounting for risk modulators.
(33)	Diagnosis and fatigue	***p =*** **0.04**	***p <*** **0.01**	Lower total reported quality of life after accounting for risk modulators.
(33)	Diagnosis and fatigue		***p =*** **0.001**	Lower school functioning accounting for risk modulators.
(33)	Diagnosis and fatigue		***p =*** **0.01**	Lower emotional functioning accounting for risk modulators.
(34)	Birthplace, education, income, stress, and treatment intensity	***p <*** **0.0001**	**β = 14.20 (3.95)**, ***p =*** **0.0005 (Foreign born)**	Higher parent post-traumatic stress.
(34)	Birthplace, education, income, stress, and treatment intensity	***p =*** **0.002**	**β = 4.35 (1.90)**, ***p =*** **0.02 (Foreign born);** **β = 4.09 (1.28)**, ***p =*** **0.0002 (US born)**	Higher rates of depression.
(39)	Family-level SES (parent education and family income)	***p <*** **0.05**	*p =* 0.25	Lower global adaptive functioning attenuated by risk modulators.
(39)	Family-level SES (parent education and family income)	***p <*** **0.01**	*p =* 0.19	Lower conceptual adaptive functioning attenuated by risk modulators.
(39)	Family-level SES (parent education and family income)	***p <*** **0.01**	*p =* 0.48	Lower social adaptive functioning attenuated by risk modulators.
(39)	Family-level SES (parent education and family income)	***p <*** **0.05**	*p =* 0.15	Lower practical adaptive functioning attenuated by risk modulators.
(42)	Age, sex, social support, family influence, PTG, depressive symptoms, treatment, self-efficacy		**OR= 0.25, 95% CI: 0.13-0.45**	Higher post-traumatic growth scores accounting for risk modulators.
NON-WHITE^*^				
(24)	Family income and caregiver education		**P=0.04**	Lower emotional quality of life accounting for risk modulators.
(33)	Diagnosis and fatigue	*p =* 0.26	***p =*** **0.04**	Lower psychosocial functioning after accounting for risk modulators.
(33)	Diagnosis and fatigue	*p =* 0.35	***p =*** **0.04**	Lower total reported quality of life after accounting for risk modulators.
(33)	Diagnosis and fatigue		***p =*** **0.01**	Lower school functioning accounting for risk modulators.
(44)	Demographic and clinical variables		***p <*** **0.01**	More positive impact of cancer in all five aspects of growth accounting for risk modulators.

*Bold denotes statistical significance with p <0.05; Reference group Non-Hispanic White or Caucasian;*

* *Listed as Other or both Non-Hispanic Black and Hispanic. SES, Socioeconomic Status; PTS, Post Traumatic Stress; QOL, Quality of Life; HR, Hazards Ratio; OR, Odd Ratio*.

In two articles, inclusion of individual characteristics and SES in multivariable modeling attenuated the significance for racial/ethnic disparities in patient-reported outcomes. Specifically, inclusion of cancer diagnosis, individual-level SES and age at study participation removed the significance for adverse mental health outcomes among non-Hispanic Black females (26). Similarly, inclusion of family-level SES removed the significance for poor global, conceptual, social, and practical adaptive functioning in Hispanic survivors (39). However, one article found that after adjusting for cancer diagnosis and fatigue symptoms, poorer psychosocial functioning and quality-of-life in minority (both non-Hispanic Black and Hispanic) survivors vs. non-Hispanic White survivors remained statistically significant (33).

### Disparities in Chronic Health Conditions

Five articles reported racial/ethnic disparities in chronic health conditions (Table 4). The type of chronic health condition disparities assessed for non-Hispanic Black survivors included vitamin-D deficiency (27), subsequent neoplasms (31), cardiovascular disorders (31), cardiovascular risks (38), and serious/life-threatening health conditions (43). The type of chronic health condition disparities assessed for Hispanic survivors included vitamin-D deficiency (27), obesity (29), subsequent neoplasm (31), endocrine condition (31). Across the articles, risk modulators included in multivariable modeling included clinical factors (diagnosis, treatment), individual characteristics (age, sex, pubertal status), individual-level SES (educational attainment, income, health insurance), family-level SES (parent educational attainment, household income), and lifestyle health risk for chronic health conditions (BMI and cardiovascular risk factors including obesity, diabetes, hypertension and dyslipidemia).

**Table 4:** Factors influencing disparities in chronic health conditions for childhood cancer survivors by race/ethnicity.

**Source**	**Risk modulators**	**Results of unadjusted models**	**Results of adjusted models**	**Interpretation of findings**
**NON-HISPANIC BLACK**				
(27)	Pubertal status	**OR = 3.11, 95% CI: 1.78–5.46**	**OR = 3.25, 95% CI: 1.83–5.78**	More likelihood of vitamin-D deficiency
(29)	Diagnosis and fatigue		OR = 2.06, 95% CI: 0.26 = 11.85, *p =* 0.436	Higher risk of obesity accounting for risk modulators.
(31)	Clinical/demographic variables		**RR = 0.6, 95% CI: 0.4–0.9**, ***p =*** **0.009**	Higher rate of subsequent neoplasms accounting for risk modulators.
(31)	Clinical/demographic variables and treatment		**RR = 0.5, 95% CI: 0.3–0.8**, ***p =*** **0.005**	Higher rate of subsequent neoplasms accounting for risk modulators.
(31)	Clinical/demographic variables, treatment, and SES (education, income, & insurance)		**RR = 0.6, 95% CI: 0.4–0.9**, ***p =*** **0.01**	Higher rate of subsequent neoplasms accounting for risk modulator.
(31)	Clinical/demographic variables, treatment, SES (education, income, & insurance), and CVRF (obesity, diabetes, hypertension, and dyslipidemia)		**RR = 0.6, 95% CI: 0.4–0.9**, ***p =*** **0.02**	Higher rate of subsequent neoplasms accounting for risk modulators.
(31)	Clinical/demographic variables		**RR = 1.9, 95% CI: 1.2–2.9**, ***p =*** **0.005**	Higher grade cardiovascular conditions accounting for risk modulators.
(31)	Clinical/demographic variables and treatment		**RR = 1.8, 95% CI: 1.1–2.7**, ***p =*** **0.01**	Higher grade cardiovascular conditions accounting for risk modulators.
(31)	Clinical/demographic variables, treatment, and SES (education, income, & insurance)		**RR = 1.6, 95% CI: 1.0–2.3**, ***p =*** **0.04**	Higher grade cardiovascular conditions accounting for risk modulators.
(38)	More or less that years of diagnosis	HR = 0.98, 95% CI: 0.52–1.86, *p =* 0.95	**HR = 1.60, 95% CI: 1.05–2.43**, ***p =*** **0.03**	Higher cardiovascular after five years accounting for risk modulators.
(43)	Treatment, diagnosis, age and gender	RR = 0.9, 95% CI: 0.7–1.2, *p =* 0.32	**RR = 1.5, 95% CI: 1.0–2.1**, ***p =*** **0.03**	Higher severity (Grade 3-4) in health conditions after accounting for risk modulators.
**HISPANIC**				
(27)	Pubertal status	**OR = 2.08, 95% CI: 1.09–3.97**	**OR = 2.14, 95% CI: 1.11–4.13**	More likelihood of vitamin-D deficiency.
(29)	Diagnosis and fatigue		**OR= 2.29, 95% CI: 1.23–4.30**	Higher risk of obesity accounting for risk modulators.
(31)	Clinical/demographic variables, treatment, SES (education, income, & insurance), and CVRF (obesity, diabetes, hypertension, and dyslipidemia)		**RR= 1.6, 95% CI: 1.2–2.3**, ***p =*** **0.005**	Higher rate of subsequent neoplasms accounting for risk modulators.
(31)	Clinical/demographic variables, treatment, and SES (education, income, & insurance)		**RR = 1.5, 95% CI: 1.1–1.2**, ***p =*** **0.01**	Increased risk for endocrine conditions accounting for risk modulators.
(31)	Clinical/demographic variables, treatment, SES (education, income, & insurance), and CVRF (obesity, diabetes, hypertension, and dyslipidemia)		**RR = 1.6, 95% CI: 1.2–2.3**, ***p =*** **0.005**	Increased risk for endocrine conditions accounting for risk modulators.

*Bold denotes statistical significance with p < 0.05; Reference group Non-Hispanic White or Caucasian. CVRF, Cardiovascular Risk Factor; SES, Socioeconomic Status; HR, Hazards Ratio; OR, Odd Ratio; RR, Relative Ratio*.

In two articles, inclusion of clinical factors, individual characteristics, and SES in the modeling attenuated the significance for racial/ethnic disparities in chronic health condition. Specifically, one article found that inclusion of clinical factors, individual characteristics, and SES factors removed the significance of disparity in subsequent neoplasms for non-Hispanic Black survivors (31). Another article suggested that inclusion of clinical and demographic factors removed the significance of the disparity in serious/life-threatening health conditions for non-Hispanic Black survivors (43). However, one article found that disparities in subsequent neoplasms and cardiovascular disorders remained significant for non-Hispanic Black survivors and disparities in subsequent neoplasms and endocrine disorders remained significant for Hispanic survivors after adjusting for clinical, cardiovascular risk, and/or individual SES factors in the modeling (31).

### Disparities in Survival Rates

Five articles reported racial/ethnic disparities in survival rates (Table 5). Type of survival outcomes assessed for non-Hispanic Black survivors included all-cause mortality (22), all-cause mortality including relative and standardized rates (31), subsequent malignancy mortality (22), risk of cardiovascular-specific death (25), and risk of any death (25). Types of survival metrics assessed for Hispanic survivors included all-cause standardized mortality rates (31). Type of survival metrics assessed for non-White survivors included hazard of death for survivors diagnosed with acute myeloid leukemia, astrocytoma, and non-astrocytoma CNS tumors (30) and mortality to incidence ratios (40). Across the articles, modulators included in multivariable modeling included clinical factors (time since cancer diagnosis, age at cancer diagnosis, cancer type), individual characteristics (age, sex), SES (educational attainment, income, health insurance), lifestyle health risk (cardiovascular risk factors such as obesity, diabetes, hypertension, dyslipidemia), neighborhood factors (census-track SES Index), and US national mortality rate (for the purpose of mortality standardization).

**Table 5:** Factors influencing disparities in survival for childhood cancer survivors by race/ethnicity.

**Source**	**Risk modulators**	**Results of unadjusted models**	**Results of adjusted models**	**Interpretation of findings**
**NON-HISPANIC BLACK**				
(22)	US mortality rates, sex, year of diagnosis		**SMR = 6.67, 95% CI: 5.84–7.59**	Higher all-cause mortality risk accounting for risk modulators.
(22)	US mortality rates, sex, year of diagnosis		**SMR = 10.72, 95% CI: 7.18–15.40**	Higher mortality risk of subsequent malignancy accounting for risk modulators.
(25)	Age at diagnosis, time since diagnosis, cancer type	**HR = 1.75, 95% CI: 1.70–1.79**	**Age 0–14 HR = 1.26, 95% CI: 1.18–1.35 Age 15–35 HR= 1.88, 95% CI: 1.83–1.93**	Higher risk of any death.
(25)	Age at diagnosis, time since diagnosis, cancer type	**HR = 2.13, 95% CI: 1.85–2.46**	Age 0–14 HR = 1.08, 95% CI: 0.62–1.89 Age 15–34 HR = 1.33, 95% CI: 0.60–2.95	Higher cardiovascular disease death attenuated by risk modulators.
(31)	Clinical/demographic variables		**RR = 1.5, 95% CI: 1.1–2.0**, ***p =*** **0.004**	Higher all-cause relative mortality rate accounting for risk modulators.
(31)	Clinical/demographic variables and treatment		**RR = 1.4, 95% CI: 1.1–1.9**, ***p =*** **0.008**	Higher all cause relative mortality rate accounting for risk modulators.
(31)	Clinical/demographic variables, treatment, and SES (education, income, & insurance)		RR = 1.0, 95% CI: 0.8–1.4, *p =* 0.88	Higher all-cause relative mortality rate accounting for risk modulators.
(31)	Clinical/demographic variables, treatment, and SES (education, income, & insurance)		**SMR = 0.6, 95% CI: 0.4–0.8**, ***p <*** **0.001**	Higher all-cause standardized mortality rate accounting for risk modulators.
(31)	Clinical/demographic variables, treatment, and SES (education, income, & insurance) and SVRF (obesity, diabetes, hypertension, and dyslipidemia)		**SMR = 0.6, 95% CI: 0.4–0.8**, ***p <*** **0.001**	Higher all-cause standardized mortality rate accounting for risk modulators.
**HISPANIC**				
(31)	Clinical/demographic variables, treatment, and SES (education, income, & insurance) and SVRF (obesity, diabetes, hypertension, and dyslipidemia)		**SMR = 0.7, 95% CI: 0.6–1.0**, ***p =*** **0.03**	Higher all-cause standardized mortality rate accounting for risk modulators.
NON-WHITE^*^				
(30)	Neighborhood-level SES index^**^	**Direct HR = 1.45, 95% CI: 1.15–1.84**, *p* < **0.01**	**Indirect HR = 1.15, 95%CI: 1.03–1.29**, ***p =*** **0.01**	Higher hazard of death for Acute Myeloid Leukemia survivors.
(30)	Neighborhood-level SES index^**^	**Direct HR = 1.80, 95% CI: 1.42–2.30**, *p* < **0.0001**	Indirect HR = 1.08, 95% CI: 0.98–1.20, *p =* 0.12	Higher hazard of death for Astrocytoma survivors attenuated by risk modulators.
(30)	Neighborhood-level SES index^**^	**Direct HR = 1.41, 95% CI: 1.11–1.78**, ***p <*** **0.01**	Indirect HR = 1.09, 95% CI; 0.97**–**1.22, *p =* 0.14	Higher hazard of death for non-astrocytoma CNS tumors attenuated by risk modulators.
(40)	None	**MIR = 27.4%**, ***p =*** **0.001**		Higher mortality to incidence without accounting for risk modulators.

*Bold denotes statistical significance with p < 0.05; Reference group Non-Hispanic White or Caucasian;*

* *Listed as other or Non-White;*

** *Tract SES Index, National Cancer Institute Census Tract-level socioeconomic status (SES) Index. CVRF, Cardiovascular Risk Factor; SES, Socioeconomic Status; HR, Hazards Ratio; OR, Odd Ratio. SMR, Standard Mortality Ration; RR, Relative Ratio; MIR, Mortality to Incidence Ratio*.

In two articles, inclusion of clinical and SES factors attenuated the significance for racial/ethnic disparities in survival outcomes. Specifically, one article found that inclusion of census-tract (i.e., neighborhood-level) SES removed the significance of death hazard for non-Hispanic Black survivors diagnosed with astrocytoma and non-astrocytoma CNS tumor, but not acute myeloid leukemia (30). Another article suggests that the adjustment individual and clinical factors removed the significance of cardiovascular-specific death for non-Hispanic Black survivors (25). However, another article found that disparities in all-cause relative mortality rates remained statistically significant for non-Hispanic Black and Hispanic survivors after adjusting for clinical factors, individual demographic and SES factors, and cardiovascular risk in the modeling (31). In addition, based on a path analysis focusing neighborhood socioeconomic determinants as the mediator, one article found significantly higher death hazard among non-White survivors of acute myeloid leukemia compared to non-Hispanic White survivors (30).

## Discussion

Compared to non-Hispanic White, non-Hispanic Black and Hispanic childhood cancer survivors suffer more from poorer health outcomes including healthcare utilization, patient-reported outcomes, chronic health conditions and survival rate. While there is an effect of race/ethnicity on health outcomes for childhood cancer survivors; there is not yet enough evidence to determine the true effect of SES across all outcomes given the cross-sectional design of previous studies. The current findings do show that embedded in race and ethnicity are a multitude of factors at the clinical (e.g., disease, treatment), individual (e.g., demographic, SES), and neighborhood (e.g., community SES) levels that may explain some of the disparities and poor health outcomes. However, the magnitude of racial/ethnic disparities changed in some but not all studies after adjusting for these risk modulators. As such, we see a complex interplay among these risk factors for health disparities. Future research is warranted to elucidate the complex associations between racial/ethnic and SES factors and health outcomes for childhood cancer survivors.

### Disparity-Specific Risk Modulators

Potential risk modulators that explained the associations between race/ethnicity and health outcomes attempted in all articles were reviewed. Risk modulators commonly reported for healthcare utilization disparity included individual-level SES (26, 28). Social support and religious importance (35–37) also explained aspects of the racial/ethnic disparities. In patient-reported outcomes, risk modulators for racial/ethnic disparities included family-level SES (23, 24, 26, 39), family dynamics (34, 42), and treatment factors (33). Particularly for Hispanic survivors, family dynamics (e.g., language spoken at home) should be further investigated as they are potentially protective factors for poor patient-reported outcomes. In chronic health conditions, most articles found that racial/ethnic disparities remained statistically significant after risk modulators (e.g., clinical factors, individual demographic and SES factors, and cardiovascular risk factors) were included in the multivariable modeling (27, 29, 31, 38, 43). It is possible that underlying biological mechanisms (e.g., inherited genetic predisposition to disease risks and epigenetic modifications due to life experiences or environmental exposures) and disadvantaged neighborhood environments may elevate disparities in chronic health conditions beyond the influence of individual SES and clinical risk. In survival rate, individual-level and neighborhood-level SES (22, 30, 31), together with age at cancer diagnosis (25, 39) and years since diagnosis, played an important role for risk facilitation (26).

Bhatia et al. argues that the “burden of morbidity and mortality [between races] is comparable because mortality is mitigated by SES” (12, 46); however, our findings suggest that the effect of SES on disparities is less straightforward. In fact, individual-level, family-level, and neighborhood-level variables may have distinct impacts on health disparities. We found that adjustment for SES increased the magnitude of disparities in some patient-reported outcomes (i.e. adverse mental health for Black females, post-traumatic stress for Hispanic parents) rather than mitigated them (23, 26). Furthermore, various sources and datasets used to quantify SES risk modulators in the analysis across studies may complicate the interpretations of findings. While the majority of the articles in our review used individual-level SES or family-level SES), one article used a validated composite SES index with seven specific indicators (proportion employed in working class occupations, proportion over 16 employed, education index, median household income, proportion below 200% poverty level, median rent and median house value) (30, 47) to capture the complex influences of different levels of SES. However, very few selected articles included neighborhood contextual factors in the analysis. In fact, neighborhood-level factors such as the built environment (e.g., green space) (48), accessibility to healthy food (49), and healthcare services (50) are increasingly considered key determinants of health outcomes for adult-onset cancer but not for pediatric cancer research. In addition, race/ethnicity-sensitive indices warrant consideration including crime-rate, incarceration, and residential segregation. The use of geospatial neighborhood metrics may provide useful information for understanding disparities in health outcomes thereby offering a more complete depiction of health disparities for childhood cancer survivors.

In addition to improving SES measurement for childhood cancer research, it is important to use a holistic and life-course approach to investigating risk of health disparities. Williams (4, 51) suggests that race is an antecedent for SES instead of a variable inside, and embedded in race and ethnicity are layered factors that may be inextricably linked. Geronimus et al., suggest the burden of physiological stress (i.e. allostatic load) of race, ethnicity, and low SES can accumulate over time (52), which in turn may link to health disparities in underserved minority breast cancer (53, 54) and general (54) populations. Cultural and familial factors can influence the impact of allostatic load (54, 55) which may explain the risk for poor patient-reported outcomes in minority survivors. Krieger (56) suggested a federal mandate to include and categorize individual-level data pertinent to racialized societal inequities and explicit justification of metrics used to categorize racial groups. Therefore, in addition to standard SES variables, the design and collection of standardized race/ethnic-specific risk modulators for childhood cancer survivors are needed.

### Racial/Ethnic Disparity-Specific Interventions

Risk modulators that substantially impact health outcomes of individual childhood cancer survivors were SES, healthcare accessibility, and health insurance. Several studies suggested that neighborhood-level SES (30), individual-level SES (26, 31) and/or family-level SES (26, 39) plays a more significant role as compared to health insurance in explaining the effects of race/ethnicity on poor health outcomes in childhood cancer survivors. In fact, a population-based study found that improving health insurance coverage alone may disproportionately benefit non-Hispanic White with lower SES rather than racial/ethnic minorities (57, 58). A more inclusive, need-based financial assistance program for individual survivors should be considered for minority survivors to reduce the risk of health disparities. In addition, the first two to three years from cancer diagnosis (25, 38, 43) and primary caregiver education background and proximity/access to care (39) were associated with elevated risk of health disparities in minority childhood cancer survivors. Therefore, healthcare systems should assess the disparity status for minority childhood cancer survivors immediately following completion of therapy and provide social support or resources to address these issues (e.g., coordinating transportation aids for minority families) toward improving follow-up care and reducing disease burden.

Our findings highlight that individual-level factors, such as culture (28, 33, 34, 37) and sex (26, 28) may contribute to racial/ethnic disparities in health outcomes. Cultural beliefs (i.e. fatalism) and gender beliefs seem relevant to health disparities in non-Hispanic Black survivors (26), while family dynamics, such as foreign-born parents experiencing greater amounts of post-traumatic stress, may impact Hispanic survivors (34, 59). In addition, minority childhood cancer survivors who had better social skills (27) and post-traumatic growth (31) were associated with better health outcomes. Therefore, it is critical to provide culture-/race-/ethnicity-/gender-specific social and emotional learning (i.e. stress prevention) interventions and diversity informed training for healthcare navigators (i.e. social workers, hospital staff, researchers, etc.). Social and emotional learning interventions that acknowledge established race-/gender-related stigma are avenues to augment resilience and provide social support and belonging.

### Racial/Ethnic Disparity in Era of Digital Health and Big Data

There is an opportunity to leverage health information technology to promote health equity for minority and underserved populations (60, 61). Emerging evidence has found that the use of eHealth and mHealth platforms can improve physiological and psychological well-being, health knowledge, and self-management skill in racial/ethnic minorities and underserved populations (62). Given the importance of visiting oncologists/primary physicians for follow-up care and maintaining healthy lifestyle among childhood cancer survivors, mHealth and eHealth technology represent the methods that may improve access to medical care (e.g., telemedicine consultation and remote lifestyle and psychological interventions), communication with healthcare providers (e.g., digital therapy and education, tailored supportive resources), and symptom monitoring and management (e.g., real-time symptom monitoring for identifying early signs of late effects) (62). However, the vast majority of current eHealth and mHealth applications are designed in the English language. Future efforts are warranted to ensure the provision of technology platforms that are multilingual and culturally and literately appropriate.

Improving medical informatics infrastructure within healthcare systems can facilitate the collection and assessment of social determinants of health data for cancer survivors on a regular-basis and integrate social determinant information into clinical decision-making process. Incorporating neighborhood-/community-level social determinant data into electronic health records (EHRs) will allow clinicians to provide tailored interventions that are clinically actionable based on the survivors' need and contextual influence. Given the big data stored in EHRs, the use of artificial intelligence analytics (e.g., machine learning and natural processing techniques) can help identify complex social determinants for individual minority survivors. Recent evidence suggests that implementation of machine learning approaches helps identify the patterns of social determinants for impaired health outcomes with superior performance compared to the use of traditional analytics (63).

### Limitations

While this scoping review provides useful information for racial/ethnic disparities in health outcomes among childhood cancer survivors, the findings should be carefully interpreted. First, race/ethnicity data from all articles were self-reported. Self-reported race/ethnicity information is often arbitrary and poorly defined (16). Furthermore, based on the available data included in the articles, we only focused on two traditionally minoritized/marginalized groups and excluded other non-White minority groups from our review. For example, American Indian childhood cancer survivors with acute lymphoblastic leukemia have lower survival rates compared to other races/ethnicities (46). Second, characteristics and patients of the survivor populations included in our review were generally homogenous. As the majority of selected studies were derived from the US-based Childhood Cancer Survivorship Study or the Surveillance Epidemiology and End Results registry, health outcome data are likely to overlap in time, collection, and patients. As mentioned in the beginning of the Results section, the percentage of minority survivors in the selected study was far lower than the percentage of the US general population. Finally, this scoping review focused on non-Hispanic Black and Hispanic health disparities, which is an emerging topic supported by current research on minoritized populations (20). In fact, the studies selected into our review did not breakdown race/ethnicity into categories beyond the three minoritized categories reported. Some articles just reported White and Other. It is critical to evaluate health disparities across more categories and intersections of races and ethnicities in the future research. It is also important to use a community-based, culture-specific participatory research design to recruit and engage racial/ethnic minorities to in childhood cancer survivorship research for better understanding the gap while also elucidating clinical interventions (64).

## Data Availability Statement

The raw data supporting the conclusions of this article will be made available by the authors, without undue reservation.

## Author Contributions

JB and I-CH: concept and design. MH and LR: administrative support. TR and TM: collection and assembly of data. TR, TM, and I-CH: data analysis and interpretation. TR and I-CH: manuscript writing. All authors editing and final approval of manuscript. All authors contributed to the article and approved the submitted version.

## Funding

The research reported in this manuscript was supported by the National Cancer Institute under award number R01CA238368 (MPIs: I-CH, JB) and V-Foundation Robin Roberts Cancer Thrivership Fund under award number DT2020-014 (MPIs: ZW, I-CH). The content is solely the responsibility of the authors and does not necessarily represent the official views of the funding agencies.

## Conflict of Interest

The authors declare that the research was conducted in the absence of any commercial or financial relationships that could be construed as a potential conflict of interest.

## Publisher's Note

All claims expressed in this article are solely those of the authors and do not necessarily represent those of their affiliated organizations, or those of the publisher, the editors and the reviewers. Any product that may be evaluated in this article, or claim that may be made by its manufacturer, is not guaranteed or endorsed by the publisher.
